# Effect of Whole-Body Vibration Training on Muscle Activation for Individuals with Knee Osteoarthritis

**DOI:** 10.1155/2021/6671390

**Published:** 2021-03-26

**Authors:** Juan Zhang, Rui Wang, Yili Zheng, Jiao Xu, Ya Wu, Xueqiang Wang

**Affiliations:** ^1^Department of Rehabilitation Medicine, Shanghai Shangti Orthopaedic Hospital, 200438 Shanghai, China; ^2^Department of Sport Rehabilitation, Shanghai University of Sport, 200438 Shanghai, China

## Abstract

Whole-body vibration (WBV) training may improve the strength of lower extremity muscles in patients with knee osteoarthritis (KOA), but the inconsistency in vibration parameters leads to differences in findings. This cross-sectional study is aimed at observing the effects of different vibration frequencies and knee flexion angles on the activation of lower extremity muscles in patients with KOA. Enrolled participants received WBV training at 0, 30, and 60° knee flexion angles with vibration frequencies of 0, 5, 10, and 20 Hz. Activation rates for vastus medialis, vastus lateralis, rectus femoris, biceps femoris, and semitendinosus in different combinations were collected through surface electromyography. The effects of frequency and angle on muscle activation rate were quantified by repeated measures ANOVA. Individual and synergistic effects of frequency and angle were also analysed. Twenty-six participants with KOA were included. Muscle activation increased with the vibration frequency in 0–20 Hz range and with knee flexion angle in 0–60° range. WBV training at 20 Hz was the most effective for knee muscle activation, and static squatting at 60° was the most suitable for WBV training. Therefore, WBV training can increase the activation rate of knee flexor and extensor muscles in patients with KOA, and the most efficient combination was 20 Hz vibration frequency and 60° knee flexion. When applying WBV to patients with KOA, individual differences and rehabilitation purposes should be considered in selecting vibration parameters and knee angle to effectively increase neuromuscular activity.

## 1. Introduction

Knee osteoarthritis (KOA) is a chronic degenerative disease characterised by the inflammation of the knee joint and surrounding soft tissues [1–3]. KOA likely occurs in women, and its prevalence increases with age. Patients often have activity pain, morning stiffness, and instability symptom which seriously affect the daily activities and quality of life [4]. Although nonsteroidal anti-inflammatory medications are widely prescribed, the high risk of side effects (gastrointestinal, renal, and cardiovascular risks) and high medical costs have limited their use [5]. Evidence-based international guideline strongly recommends exercise as a nonsurgical therapy for KOA management [6]. Several systematic reviews reported that resistance training has a moderate effect on pain and physical function for patients with KOA [7, 8]. Meta-analyses revealed the increasing overall risk of developing symptomatic KOA for people with knee extensor muscle weakness [9, 10]. Weak lower knee extensor strength would also affect patients' stability in action and is associated with functional deterioration [10]. Therefore, strength and stability training of lower extremities is regarded as one of the cores of exercise therapy for KOA.

Whole-body vibration therapy (WBV) is an effective neuromuscular training that uses mechanical vibration with different frequencies to stimulate repeated muscle contractions to improve muscle function and proprioception [11]. Under optional magnitude, frequency, and duration [12, 13], WBV is more suitable for KOA than resistance training and is safer for individuals who cannot perform high-intensity exercise. WBV is widely used in different clinical studies, such as those focusing on osteoporosis [14], fibromyalgia [15], and KOA [16, 17].

The effectiveness of WBV on pain, muscle strength, and proprioception for patients with KOA is controversial. A meta-analysis showed that WBV does not induce a substantial difference in pain intensity and self-reported status compared with other exercises, such as the 6-minute walking test and time up and go test [18]. Another review showed that WBV training enhances functional performance and reduces pain in patients with KOA [19]. One randomised controlled trial concluded that a 4-month WBV can enhance jumping power in young adults, suggesting the occurrence of neuromuscular adaptation to the vibration stimulus [20]. Pamukoff et al. [21] found that WBV and local muscle vibration enhance the quadricep strength in healthy adults, but Segal et al. [22] reported that a 12-week WBV exercise does not remarkably improve the muscle strength of lower extremities for patients with KOA. Inconsistencies in the parameters of the WBV intervention scheme are one of the important factors that contribute to the difference in research results.

Most studies used medium-to-high vibration frequencies (25–45 Hz) with varying effectiveness on muscle strength, proprioception, and balance [23, 24]. Differences in knee angle during exercise program may also influence the outcomes [25]. Therefore, the present work is aimed at exploring the effects of different low vibration frequencies and knee flexion angles on the muscle activation of patients with KOA who received WBV. The primary hypotheses were as follows: (1) in the WBV low-frequency group (0–20 Hz), the neuromuscular activity in the lower extremities of patients with KOA is progressively induced by the increasing frequency, and (2) a synergistic relationship occurs between the effects of knee angle and vibration frequency on muscle activation.

## 2. Methods

### 2.1. Design

This study was a cross-sectional experiment involving female patients with KOA. The study was approved by the Ethics Committee of the Shanghai University of Sport and was registered at the Chinese clinical trial registry (ChiCTR-IOR-16009234). All included participants were required to complete 12 vibration regimens, and the muscle activities of their low extremities were collected by using surface electromyography (EMG) equipment. The effect size was set at 0.49 [26], and the primary outcome was muscle activation. Repeated measures ANOVA was used in the G∗power software with an alpha of 0.05, power of 0.95, and number of measurements of 12. Considering 25% of attrition rate, at least 24 participants were required.

### 2.2. Participants

All potential participants were recruited from three streets (Huangxing Street, Yinxing Street, and Ouyang Street) in Yangpu District, Shanghai. Twenty-six women with KOA participated aged 50–70 years who met the classification criteria of the American Rheumatism Association for KOA and had radiographic evidence of KOA in one or both sides were included. [27] All participants reported pain for more than 3 months with different disease courses and no neurological illness. Exclusion criteria were as follows: had a history of knee injury in the past six months; experienced acute symptomatic arthritis; had pain intensity greater than seven as rated by a visual analogue scale which is a 100 mm line marked “no pain” and “worst pain” at both ends, and the score is measured from zero to the patient's mark [28]; had other conditions (such as osteomyelitis, tuberculosis, and tumour) that affect their walking function; had a contraindication to exercise; and exhibited cognitive impairment. Each participant signed a written informed consent prior to baseline assessment.

### 2.3. Procedure

The study was completed in the Rehabilitation Center of Sports Medicine of Shanghai University of Sport. Baseline demographic characteristics, such as age, body mass index (BMI)—body weight normalized by height squared (kg/m^2^) [29], range of motion (ROM) of knee joints by using a mechanical inclinometer [30], and Western Ontario and McMasters Arthritis Index (WOMAC) [31], were collected for all participants. Prior to WBV training, they were required to wear electrodes to complete the maximal voluntary contraction (MVC) tests of the extensor and flexor muscles of the knee. The muscles tested were the following: rectus femoris (RF), the midpoint of the line between the anterior inferior iliac spine and the upper margin of the patella; vastus lateralis (VL), the lower third of the line between the outer margin of the patella and the greater trochanter of the femur; vastus medialis (VM), the point was located 3 cm above the internal upper corner of the patella and then 2 cm inward; semitendinosus (S), the lower third of the line between the ischium tubercle and the medial upper end of the tibia; and biceps femoris (BF), the midpoint of the line between the ischium tubercle and the medial upper end of the tibia. The skin needed to be cleaned to improve the electrical conductivity of the skin before placing the sensors. The MVC test was conducted as follows. The participants slowly bend or stretch their knees against external resistance applied by the tester. After the muscle had reached its maximum contraction force, contraction was sustained for another 5 seconds. The sensors collected the electromyographic signals produced by each muscle during its maximum contraction. MyoResearch XP Master Software (Version 1.07.17) was used for data processing.

After resting for 5 minutes, the participants stood on the WBV platform (AV-001, BODYGREEN, Taiwan, China) with bare feet shoulder-width apart and completed static squats at 0°, 30°, and 60° of knee joint flexion with 10 seconds for each squat and a 1-minute rest (Figure 1). Surface EMG equipment based on DTS (Noraxon Inc., Scottsdale, USA) was used to collect data on muscle activity, and the sampling frequency was 1500 Hz. The parameters of WBV were set as follows: the amplitude was 1.5 mm, the vibration type was vertical vibration, and the frequency was set to 0, 5, 10, and 20 Hz for each angle. The bending angle and vibration frequency were designated as independent variables. Each participant should complete 12 combinations with random angles and frequencies during the test.

### 2.4. Outcomes

Time domain analysis can calculate characteristic parameters, such as root mean square (RMS), which reflect the changes of the EMG signal in time. A high RMS of EMG indicates a high muscle activation rate [32]. The maximum RMS in the MVC was used for myoelectric standardized analysis. Muscle activity in different combinations was represented by muscle activation rate (EMG%_MVC_), which is equal to the actual RMS divided by the maximum RMS of MVC times 100%.

### 2.5. Statistical Analysis

All data were presented as means ± standard. IBM SPSS Statistics 20.0 software (SPSS Inc., Chicago, USA) and Microsoft Excel 2016 were used for data analysis. The EMG%_MVC_ of each muscle under different conditions was statistically analysed using the two-factor (frequency∗angle) repeated measures ANOVA. This study determined whether frequency or angle has main effects and whether they interact with each other. When the two factors had significant interaction, the influence of one factor on EMG%_MVC_ at different levels of the other factor was analysed successively. If the two factors had a significant main effect, then Bonferroni adjustments were used for post hoc analysis. A significant level was set as *P* < 0.05.

## 3. Results

Twenty-six women with KOA with a mean age of 61.4 ± 5.3 years and a mean BMI of 23.9 ± 3.0 kg/m^2^ were enrolled. All participants had a 116.4° ± 12.5° ROM of the knee joint with mild-to-moderate pain (visual analogue scale score of 2.82 ± 2.41) and WOMAC score of 25.86 ± 34.64. The flexion angle and vibration frequency had significant interaction on the activation of VM, but not on VL, RF, S, and BF (Table 1).

At 0 and 30° knee angles, the vibration frequency induced a significant difference on VM activation, and the EMG%_MVC_ increased with the frequency. At 20 Hz, the EMG%_MVC_ of VM was the highest. No significant difference was observed when the angle was 60°. At 0, 5, 10, and 20 Hz, the angle induced a significant difference on VM activation, and the EMG%_MVC_ of VM increased with the angle. At 60° knee angle, the EMG%_MVC_ of VM was the highest (Table 2). Various vibration frequencies induced significant differences on the EMG%_MVC_ of RF, S, and BF, but not on that of VL (Table 3). Various angles induced significant differences on the EMG%_MVC_ of VL, RF, and BF but not on that of S (Table 4).

Under different vibration frequencies, the EMG%_MVC_ of VM was significantly different among the three angles. At 0° knee joint, significant differences on the EMG%_MVC_ of VM were observed between 0 and 20 Hz, 5 and 20 Hz, and 10 and 20 Hz. At 30° of the knee joint, significant differences on the EMG%_MVC_ of VM were observed between 0 and 10 Hz and 0 and 20 Hz. No statistical differences for the EMG%_MVC_ of VM were found under other combination conditions. Given the lack of interaction between the effects of frequency and angle on the EMG%_MVC_ of VL, RF, S, and BF, the individual influences of these two factors were subsequently analysed. Significant differences on the EMG%_MVC_ values were found as follows: for VL, between 0 and 30°, 0 and 60°, and 30 and 60°; for RF, between 0 and 20 Hz, 5 and 10 Hz and 5 and 20 Hz, 10 and 20 Hz, and 0° and 60°; for S, between 0 and 5 Hz, 0 and 10 Hz, 0 and 20 Hz, 5 and 10 Hz, 5 and 20 Hz, and 10 and 20 Hz; and for BF, between 0 and 10 Hz, 0 and 20 Hz, 5 and 10 Hz, 5 and 20 Hz, and 10 and 20 Hz and between 0 and 30°, 0 and 60°, and 30 and 60°.

## 4. Discussion

The results showed that in the range of 0-20 Hz, the activation rates of muscles, except for VL, gradually increased with vibration frequency, consistent with the first hypothesis. And the neuromuscular activity was highest at 20 Hz, regardless of the knee angle. However, only the knee angle and WBV frequency had significant interaction on the EMG%_MVC_ of VM. The EMG%_MVC_ values of VM, RF, and BF were significantly different at various knee angles. All tested muscles had the highest activation rate at the combination of 20 Hz and 60°, and WBV significantly increased muscle activity. Therefore, if an individual with KOA does not have a large ROM of the knee joint, then muscle activation can be increased by appropriately increasing the WBV frequency. This finding is also applicable to patients who are unable to tolerate high vibration frequency; an appropriate increase in knee angle can achieve a comparable muscle activation. Therefore, individual differences and training purposes should be considered when choosing a WBV scheme.

The results showed that a high WBV intensity at a certain frequency and angle is associated with great EMG amplitude of lower limb muscles, and this finding is generally consistent with other studies [33–37]. The increase in EMG amplitude indicates that WBV training can enhance the motor nerve regulation function, which is reflected in the change of motor unit recruitment form and quantity [38, 39]. In muscle contraction, the body's protective mechanism controls the ability of some motor units to mobilise. Meanwhile, other units are in a state of potential. In a vibrating environment, the produced stimulus changes the length of the fusiform muscle, which activates the excitability of the muscle spindle and causes muscle fibre contraction [40]. Thus, vibration increases the extent of maximum recruitment for motor units under active muscular contraction, such as in static squatting. Vibration also leads to the high stimulation of muscle mechanoreceptors accompanied by an increase in tension. This response is similar to the tonic vibration reflex, the involuntary reflex contraction of muscles caused by vibration stimulation [41, 42]. Synchronised discharges of motor units subsequently lead to a high contraction force. The acceleration produced by vibration stimulation is another possible reason for the increase in motor unit recruitment, which allows a surge in muscle strength under small motion load [38, 43]. Stretch-shortening cycle training is a method of immediate centripetal contraction after centrifugal contraction [44]. This activity stimulates the neuromuscular system through the stretch reflex to generate additional muscle activity and power. WBV training functions similarly to the physiological mechanism of a stretch-shortening cycle; however, the former is a closed chain movement that avoids the impact of the body on the ground to reduce the risk of sports injuries. Hence, WBV is suitable for the elderly who cannot perform resistance training [37].

During WBV, the constant changes in an individual's load consequently alter the nervous system with the vibration stimulation. Therefore, this training improves the responsiveness of the neuroregulatory system. Osawa et al. [33] found that WBV could improve knee extension muscle strength and countermovement jump. The present study also found that WBV increased the activation of BF and S muscles under either exercise regimen. This finding indicated that vibration can enhance the activation of agonistic and antagonistic muscles and the coordination of nervous and muscle systems, thus improving the reaction ability of knee flexor and extensor muscles. Bolgla et al. [45] pointed out that closed chain action training effectively activates VM. Irish et al. [46] studied the activation characteristics of VL and VM during closed and open chain movements and found that their activation ratio during closed chain movement was higher than that of the knee extensor trained under the seated position with no weight. Therefore, the closed chain motion can balance the power of VL and VM. In patients with KOA, the activation of VM is less than of VL, resulting in the poor stability of the knee joint. Therefore, closed chain movements, such as double foot squats, can increase the synchronous activation of VL and VM and exhibit an advantage in VM activation.

The frequency range of the WBV device is between 0 and 50 Hz. The results showed that except for VL, all the muscles had the greatest EMG amplitude under the stimulation of 20 Hz vibration regardless of knee angle. Mester et al. [38] reported that quadriceps femoris activation increases with vibration frequency (5 Hz to 24 Hz). Cardinale and Lim [41] confirmed that 30 Hz induces greater EMG amplitude of VL compared with 40 and 50 Hz. Pollock et al. [47] found that increasing the frequency of WBV (5–30 Hz, 2.5–5.5 mm) also increases the EMG amplitude of various leg muscles by 5% to 50% in 12 healthy adults. However, other studies reported that WBV at 30–45 Hz and 2–5 mm amplitudes can lead to leg muscle activity up to 34.5% in young adults [26, 41]. The above studies did not use filtering and possibly overestimated the muscle activity.

The contact area between the patella and the femur is the largest when the knee angle is between 60 and 90°. This condition may increase the symptoms of joint pain. Hence, knee flexion must be maintained below 60° during static squat training. The present results were consistent with Roelants et al., who stated that muscle activation rate increases with knee flexion angle and varies between 12.6% and 82.4% during WBV training [26]. When the muscle is stretched, the sensitivity of the muscle spindle increases. BF controls the thigh extension and knee flexion. In the current study, the EMG amplitude of BF increased with the knee angle. This phenomenon may be because of the increased sensitivity of BF's muscle spindle and the increased activity of motor neurons, thus leading to the enhanced recruitment of motor units. However, no significant difference in the activation rate of S was observed under different angles. S may have reached a high activation level within the flexion range. Additionally, vibration frequency, amplitude, joint angle, vibration type, and other factors may lead to different results.

In the current study, only the frequency and angle showed a significant interaction on the VM. The EMG amplitude of the VM at 60° was higher than that at 30°, which was higher than that at 0°. The increase in muscle length is the primary cause of the vibration effect [42] . Avelar et al. [48] compared the influence of knee flexion at 90° and 60° on muscle activation and found a positive correlation between them. In semisquats, the quadriceps need to generate additional force against resistance. The sensitivity of motor afferent nerves can be increased when vibration stimulation is introduced [42]. Therefore, an increase in the knee flexion angle can improve VM activation.

This study analysed the differences between muscle activation rates of knee flexor and extensor muscles in patients with KOA under various combinations of knee flexor angles and vibration frequencies, and the results provided objective evidence for the guidance of WBV training for patients with KOA. There also had some limitations. Firstly, the study had a cross-sectional design and lacked efficacy comparisons. Whether this program can effectively improve muscle function after long-term WBV training remains to be further investigated. Secondly, only the effects of low-frequency vibration and angle of knee flexion on muscle activation were analysed. Factors such as vibrator type, amplitude, and individual posture can influence the effect of WBV on muscle activation [49]. The enhancement of muscle strength begins with neural adaptation and then changes in morphology. Future studies can use elastic imaging, ultrasound, and other technologies to evaluate muscles and further improve biomechanical, biochemical, and physiological correlation analyses to learn the effectiveness of WBV on muscles.

In conclusion, WBV training can increase activation rates of knee flexor and extensor muscles in patients with KOA. Muscle activation increased with the vibration frequency in the 0–20 Hz range and with the knee flexion angle in the 0–60° range. WBV training at 20 Hz was the most effective for activation of knee flexor and extensor muscles in patients with KOA, and static squatting at 60° was the most suitable for WBV training.

## Figures and Tables

**Figure 1:** Three postures on the whole-body vibration training platform: (a) 0° knee flexion; (b) 30° knee flexion; (c) 60° knee flexion.

**Table 1:** Synergistic effects of frequency and angle on the EMG%_MVC_ of VM, VL, RF, S, and BF.

Muscle	Frequency	0°	30°	60°	*F*	*P*	Partial *η*^2^
VM	0 Hz	3.4 ± 0.5	21.6 ± 2.1	39.4 ± 3.2	4.586	0.017	0.096
	5 Hz	3.2 ± 0.6	24.6 ± 1.9	40.4 ± 3.2			
	10 Hz	4.8 ± 0.7	27.3 ± 2.4	40.1 ± 3.3			
	20 Hz	12.3 ± 2.9	33.1 ± 3.8	42.4 ± 3.1			

VL	0 Hz	4.8 ± 0.9	25.6 ± 2.3	43.6 ± 4.9	0.849	0.363	0.019
	5 Hz	4.3 ± 0.8	28.9 ± 2.8	44.3 ± 4.5			
	10 Hz	5.0 ± 1.0	28.7 ± 2.9	45.3 ± 4.7			
	20 Hz	13.1 ± 2.5	34.9 ± 4.0	92.5 ± 44.5			

RF	0 Hz	3.9 ± 0.6	14.3 ± 1.7	23.3 ± 3.4	0.982	0.389	0.022
	5 Hz	3.6 ± 0.6	16.4 ± 2.2	24.3 ± 3.2			
	10 Hz	5.5 ± 0.9	17.6 ± 2.2	25.0 ± 3.4			
	20 Hz	14.4 ± 2.1	24.4 ± 3.1	30.9 ± 4.6			

S	0 Hz	5.7 ± 1.5	5.0 ± 1.1	7.1 ± 1.7	0.882	0.437	0.020
	5 Hz	5.5 ± 1.0	5.9 ± 1.3	6.9 ± 1.7			
	10 Hz	7.0 ± 1.3	6.8 ± 1.3	8.1 ± 2.0			
	20 Hz	12.6 ± 2.5	15.4 ± 3.3	15.2 ± 3.2			

BF	0 Hz	1.3 ± 0.2	10.5 ± 1.9	18.2 ± 2.3	0.907	0.407	0.021
	5 Hz	1.3 ± 0.2	11.7 ± 1.7	18.9 ± 2.4			
	10 Hz	2.2 ± 0.3	12.6 ± 1.6	18.7 ± 2.4			
	20 Hz	5.7 ± 0.6	15.3 ± 2.0	20.8 ± 2.7			

Abbreviations: EMG%_MVC_: muscle activation rate; VM: vastus medialis; VL: vastus lateralis; RF: rectus femoris; S: semitendinosus; BF: biceps femoris.

**Table 2:** Main effects of frequency (or angle) on the EMG%_MVC_ of VM under different angles (or different frequencies).

Parameters		95% CI	*F*	*P*	Partial *η*^2^
0°	0 Hz	2.3-4.5	8.914	0.03	0.172
	5 Hz	2.2-4.3			
	10 Hz	3.3-6.2			
	20 Hz	6.5-18.1			

30°	0 Hz	17.3-25.9	8.151	0.02	0.159
	5 Hz	20.7-28.4			
	10 Hz	22.6-32.1			
	20 Hz	25.5-40.7			

60°	0 Hz	33.0-45.8	1.322	0.272	0.03
	5 Hz	33.9-46.9			
	10 Hz	33.4-46.9			
	20 Hz	33.0-45.8			

0 Hz	0°	2.3-4.5	106.861	<0.001	0.713
	30°	17.3-25.9			
	60°	33.0-45.8			

5 Hz	0°	2.2-4.3	120.733	<0.001	0.737
	30°	20.7-28.4			
	60°	33.9-46.9			

10 Hz	0°	3.3-6.2	98.255	<0.001	0.696
	30°	22.6-32.1			
	60°	33.4-46.9			

20 Hz	0°	6.5-18.1	56.058	<0.001	0.566
	30°	25.5-40.7			
	60°	33.0-45.8			

Abbreviations: EMG%_MVC_: muscle activation rate; VM: vastus medialis; CI: confidence interval.

**Table 3:** Main effects of frequency on the EMG%_MVC_ of VL, RF, S, and BF.

Muscle	Frequency	Means ± standard	95% CI	*F*	*P*	Partial *η*^2^
VL	0 Hz	24.1 ± 2.3	20.2-2.3	2.151	0.150	0.048
	5 Hz	25.8 ± 2.5	21.3-30.3			
	10 Hz	26.3 ± 2.6	17.5-24.2			
	20 Hz	46.8 ± 15.1	22.3-8.2			

RF	0 Hz	13.9 ± 1.7	11.0-16.7	22.572	<0.001	0.344
	5 Hz	14.8 ± 1.7	11.8-17.8			
	10 Hz	16.0 ± 1.8	13.0-19.1			
	20 Hz	23.3 ± 2.3	19.2-27.3			

S	0 Hz	6.0 ± 0.8	4.3-7.6	16.077	<0.001	0.272
	5 Hz	8.1 ± 0.8	6.5-9.7			
	10 Hz	10.3 ± 0.9	6.5-11.2			
	20 Hz	14.4 ± 1.7	11.0-17.8			

BF	0 Hz	10.0 ± 1.3	7.7-12.3	8.573	0.002	0.048
	5 Hz	10.6 ± 1.3	8.3-12.9			
	10 Hz	11.2 ± 1.3	8.9-13.4			
	20 Hz	13.9 ± 1.4	11.5-16.4			

Abbreviations: EMG%_MVC_: muscle activation rate; VL: vastus lateralis; RF: rectus femoris; S: semitendinosus; BF: biceps femoris; CI: confidence interval.

**Table 4:** Main effects of angle on the EMG%_MVC_ of VL, RF, S, and BF.

Muscle	Angle	Means ± standard	95% CI	*F*	*P*	Partial *η*^2^
VL	0°	6.8 ± 0.8	5.3-8.3	12.603	0.001	0.227
	30°	29.5 ± 1.5	26.5-32.5			
	60°	56.4 ± 11.3	34.1-78.8			

RF	0°	6.8 ± 0.7	5.5-8.2	33.690	<0.001	0.439
	30°	18.3 ± 1.2	15.8-20.6			
	60°	26.0 ± 1.8	22.3-29.5			

S	0°	7.7 ± 0.9	6.0-9.4	1.132	0.304	0.026
	30°	8.5 ± 1.0	6.3-10.3			
	60°	9.7 ± 1.2	7.1-11.6			

BF	0°	2.6 ± 0.3	2.1-3.1	54.930	<0.001	0.561
	30°	12.6 ± 1.7	10.8-14.4			
	60°	19.2 ± 2.3	16.8-21.6			

Abbreviations: EMG%_MVC_: muscle activation rate; VL: vastus lateralis; RF: rectus femoris; S: semitendinosus; BF: biceps femoris; CI: confidence interval.

## Data Availability

The data that support the findings of this study are available from the corresponding author upon reasonable request.
